# An Exploration of the Environment, Composition, and Transmission of the Development of Local Theater and Music in the Natural Environment and Folklore Activities of Tea Picking

**DOI:** 10.1155/2022/9491745

**Published:** 2022-07-12

**Authors:** Na Zhang

**Affiliations:** School of Music and Dance, Yichun University, Yichun 336000, Jiangxi, China

## Abstract

The spread and urbanization of modern culture have led to a crisis in the development and inheritance of traditional culture, coupled with the limitations of traditional drama itself, and local opera has gradually disappeared from the daily life of the local people. Through the analysis of the tea opera cases and the development environment and inheritance of local operas, the paper tries to solve the inheritance dilemma it faces and provides a new perspective and demonstration for the development and inheritance research of Bobai Jinan tea Opera, which is of great significance to the development and propaganda of traditional Chinese culture.

## 1. Introduction

The tea opera is a theatrical presentation of the national culture of tea picking in the mountains; through the performance of the actors, the audience is put into the tea-picking activity, projecting the natural environment of tea picking and deriving the psychology of memorialising and caring for the natural environment of the tea mountains.

Opera, as the name suggests, is a form of drama that combines poetry, music, dance, and other arts. As a local art generated by the history of a specific region, the inheritance and development of local opera are inseparable from the cultural ecology of the specific region that nurtured its growth. Local opera originated from the regional customs in the farming society, and it has developed and matured in the practice of public life and then has a complete script and performance program [1]. The reform and opening up that started in the 1980s pushed Chinese society into a rapid modernization process. Modern civilization has changed people's daily life with incomparable penetrability, leading to the decline of traditional culture and local opera art. Particularly due to the fact that “the market economy has changed the traditional cultural ecology, the spread of modern culture has led to a crisis of traditional cultural identity, and urbanization has accelerated the disintegration of the original cultural space” coupled with the limitations of traditional drama itself, the popular regions, and performances of local dramas all over the country [2]. They have been greatly reduced, and local operas have gradually faded out of the daily life of the local people. Many local operas have disappeared from the daily life of the public and become unreproducible historical memories [3]. Many local operas are in an endangered state and have almost fallen into an irreversible overall inheritance crisis [4]. The art of opera was very popular in the early twentieth century, such as Peking Opera, Kunqu Opera, and some local operas (Qin Opera, Cantonese Opera, Jin Opera, Henan Opera, and Yue Opera) [5].

After the founding of New China, the development of local opera was unprecedentedly prosperous, and some small operas were also born. Nowadays, Chinese opera has entered a stage of slow development, in which there are objective external and developmental factors, including the market occupation of the new culture, and the content of this paper is too outdated, but the author believes that it is necessary to find problems from oneself and to dig deep into the cultural value of local opera because cultural things will be in any era [6]. There is market demand, and the presentation of culture is the key issue. According to data research, the ways that people understand traditional culture mainly include several ways shown in Figure 1. Faced with the development of local operas today, we must first look at how much we have inherited or whether it is that “flavor;” secondly, we should think about how to develop and whether we have found a way for the development of this type of opera because each type of opera has certain differences [7]. There are both commonalities and differences in the problems of the local opera, so a specific analysis should be carried out according to the problems of the local opera [8]. Chinese opera art is composed of many local operas such as Peking Opera and Kunqu Opera. There are 348 local operas in existence [9]. Local opera is another manifestation of regional culture and local ethnic culture. Sex has become the cultural characteristic of local opera. In the era of rapid development, the pace of development of the art of opera has become slow. This does not mean that the art of opera is outdated, nor is it that the audience does not like opera, but to find problems fundamentally, inherit and retain classic and excellent content, and realize development with the times [10]. This paper puts forward the author's research on the inheritance and development of local opera in recent years and uses examples to illustrate the effective measures that can be taken for the protection, inheritance, and development of folk art [11].

Local opera is a local art bred by the local culture of a certain region during the farming society and has been inherited and developed in the survival practice of its creators. After entering the modern society, with the gradual disintegration of the local field on which survival depends, local opera has fallen into an increasingly serious crisis of inheritance. Through the practical logic analysis of the environment, composition, and inheritance of local opera and music development, it tries to solve the inheritance dilemma it faces and supplements new perspectives and interpretation paradigms for the inheritance research of local opera.

Drama originated from folk sacrifices in ancient times. As early as the pre-Qin period, there were witch songs and dances that entertained both gods and people [12]. It lasted for thousands of years and formed local dramas with dialects, local customs, and national characteristics as important features. Since the reform and opening up, the party and the government have invested a lot of money and strength in the prosperity and development of local opera art, and local governments have also introduced some relevant protection measures so that local opera and national art have a new look after the “Cultural Revolution.” However, with the rapid development of society and the influx of Western culture, local operas with dialect as an important feature have encountered different degrees of crisis in the market competition. According to China Culture News, on May 12, 2011, there were 16 Beijing and Kunqu Opera troupes that retained the nature of public institutions, and there used to be more than 300 kinds of local operas, but now only 13 have survived, which is obviously too few [13]. When Chairman Mao Zedong formulated the eight-character policy for the party's opera work, he wrote “let a hundred flowers bloom” before “introduce the old and bring forth the new,” which can be understood as a special emphasis on protecting the diversity of ethnic folk opera and encouraging them to achieve common prosperity through innovation and free competition. Only when Peking Opera, Kunqu Opera, and other local operas can be protected and have the opportunity to survive and develop is the true blooming of Chinese opera. Shaanxi is one of the regions with a wide variety of local operas in China. In addition to the widely popular Qin Opera, Meihu, Wanwan Opera, Shangluo Huagu, and other major operas, there are also very original ones, including Tongzhou Bangzi and Huayin Lao Opera. There are authentic Shaanxi local small operas such as Fuping A Palace Opera, Chondboard Opera, Han Diao Erhuang, Huaxian Shadow Play, Heyang Line Opera, Xinchi Dance Opera, Storytelling in Northern Shaanxi, and Xi'an Drum Music. In the late 1980s, Shaanxi local opera was under the impact of modern and powerful cultures such as film and television and pop music. There are nearly 30 local operas in the province; only Qin Opera, Meihu, Wanwan Opera, Shangluo Huagu, Jin Opera, and other operas have long-term performances; with the disintegration or dissolution of troupes in other places, the operas are almost on the verge of extinction. The only performances are only fragmented performances and opera solo performances by actors in groups of three or five during festivals, weddings and festivals, temple fairs, and sacrifices. Since the beginning of the twenty-first century, with the launch of the national intangible cultural heritage protection project, a number of local operas such as Qin Opera, Han Diaojie, and Heyang Dance Opera have been included in the national and Shaanxi provincial intangible cultural heritage protection lists [14], as shown in Table 1.

With the national and provincial intangible cultural protection efforts and investment funds increasing and increasing year by year, local opera, which was almost dead, has gradually survived and has developed to a certain extent. Especially in recent years, Shaanxi's economy has entered the fast lane of rapid development, and local operas have also appeared vigorously along with the economic development [15].

High-level stage artworks and performances have also moved from the original performances of Chinese New Year and festivals, worship of gods, weddings, funerals, and marriages to mainstream performances in the city. For example, the Zhidan County Song and Dance Troupe, established in 2007, has successively launched a series of themes such as “Ode to the Red City,” “Love in the Red City,” “Hanging the Red Light,” and “Orchid Flower” with the strong support of the county party committee and the county government. Outstanding stage artworks with bright, broad themes, diverse styles, and strong artistic appeal. In particular, the large-scale Xintianyou song and dance drama “Hanging the Red Light” and “Orchid Flower” in northern Shaanxi achieved great success in Zhidan, Yan'an, Xi'an, Nanjing, and Beijing and won unanimous praise from national, provincial, and municipal leaders and all sectors of society. “Hanging the Red Lantern” participated in the “China International Youth Art Week,” the 5th Shaanxi Provincial Arts Festival, and the 1st Shaanxi Provincial Farmers' Art Festival, which was a large-scale cultural event to welcome the Olympics. The Shaanxi Provincial Arts Festival Organization Award, Repertoire Award, Screenwriter Award, Director Award, Outstanding Performance Award, Outstanding Stage Design Award, Lighting Award, and Costume Award. After the successful performance of “Orchid Flower” in China, the province, the city, and the county, it participated in the 6th Shaanxi Arts Festival in October this year and won the Outstanding Play Award, Outstanding Performance Award, and Outstanding Stage Design Award. The dance “The Man in Northern Shaanxi” won the second prize in the 9th National Dance Competition. The sketch “The Fragrance of Fruit Flowers” won the Outstanding Performance Award in the 2nd Shaanxi Provincial Small Opera Sketch Competition in 2008 and the Outstanding Play Award and Director Award in the First Shaanxi Provincial Farmers Art Festival. “Hongdu Group” won the second prize in the 2nd Shaanxi Provincial Folk Song Competition in Northern Shaanxi Province and the first prize in the Yan'an City Shaanbei Folk Song Competition. Secondly, Zhidan County Song and Dance Troupe can dedicate a party to cadres, workers, and urban residents every month and truly become a mainstream performance group in the city. Jia Pingwa, a famous writer from Shaanxi, loves Qin Opera. In his prose “Qin Opera,” written in the 1980s, he described the love of Shaanxi people for Qin Opera, especially the obsession of rural people with Qin Opera, the simple and honest farmers. The image is vivid and vivid, Qin Feng and Qin Yun are so natural and harmonious, the Huangtian Houtu of the eight hundred miles of Qinchuan interprets the joys, sorrows, and joys of the Qin people, and the Qin Opera is their stage, in a hearty mood. However, there is really not much that has been passed down now. As far as Zhidan County People's Troupe is concerned, it was established in December 1951 and has been popular for more than 50 years. It has passed down generations to cultivate national-level actors and provincial-level excellent plays. For example, “Dou E's Injustice,” “Three Drops of Blood,” “Golden Hairpin,” “Civefish for the Prince,” “The Case of Gu Mei,” “The Red Account,” “Wangjiawan People,” and so on are provincial award-winning plays. Now it has disappeared. The troupe was also forced to disband in 2007.

The “2018 Douyin Big Data Report” (hereinafter referred to as the “Report”) shows that Huangmei Opera in Anhui has become the most popular local opera, while Henan Henan Opera, Shaanxi Qin Opera, Hunan Huagu Opera, and Zhejiang Kunqu Opera are widely spread on Douyin, occupying the top five local operas (shown in Figure 2).

In the past two years, with the continuous popularity of short videos, there are also local dramas that have opened up new online spaces. Take Taikang Taoist drama as an example. It is understood that the troupe currently has 27 Douyin accounts, 12 Kuaishou accounts, and 18 Volcano small video accounts. The video content is rehearsed and performed daily. For example, the troupe's actress Yanling Li, a Yu opera singer who is active in the field of short videos, the three short video accounts have released a total of 2,372 videos, with more than 150,000 fans and nearly 400,000 likes. In addition, there are 6 actors with more than 10,000 fans, and other actors also have different numbers of fans, forming the influence of Taikang Taoist drama on the Internet. Taking the volcano video as an example, the statistics are as follows, as shown in Table 2.

## 2. Traditional Local Opera

### 2.1. The Local Character

Most of the local operas in our country were produced and developed in the farming society, and the interweaving of agricultural economy and rural humanities created the locality of local operas in terms of content, subject matter, theme, and style. Therefore, the themes of local opera performances are close to the daily life of the local people, and the life stories of talented and beautiful women, elders and children, benevolent filial piety, and heroes are used to promote the moral norms of punishing evil and promoting good in civil society. The plot is simple, the theme is clear, it is easy to understand, and it is mainly based on comedy, which combines reasoning with music, brings people the joy and teaching of gentle wind and drizzle, and is deeply loved by the local people [16].

The important thing is that the local life rooted in local opera is the life model of rural villagers, and the folk art it nurtures is not affected by the strict standardization of mainstream culture, thus achieving the simple and beautiful local characteristics and free and flexible artistic style of local opera. Therefore, local opera has a strong taste of local culture, expresses the lifestyle of rural people, and interprets their simple thoughts and emotions with tunes that are consistent with the regional customs. It is a typical “grassroots” art. For example, Kunqu Opera retains the folk art characteristics of Southern Opera, and the performance is not restricted, free and lively, and strong in randomness. Cantonese Opera and Niu Niang Opera in Guangdong and Guangxi are both known for their “exploding belly,” and “the play is in the belly, and it is improvised to sing”; that is, the actors improvise according to the theme of the play, with a greater degree of freedom. The plot of the local drama is simple, and the performance sets, props, and soundtracks are relatively simple. Three or five actors can hang a curtain on the spot to act, which is very suitable for the simple aesthetic and entertainment needs of farmers. In terms of expression, the dialects and accents used in local operas have a strong local flavor, the lyrics and dialogues are colloquial, and the vocals are clear and lively. The tone used in any local opera is consistent with the dialect, and generally, it can only be sung in its regional dialect, reflecting the musical beauty of this dialect. It can be seen that the generation, development, and derivation of local opera all depend on the long-term infiltration of regional culture, and the performance program close to the life of farmers interprets the life world of farmers and enriches the daily life of farmers. Therefore, local opera has a strong local character and is the folk culture with the most local complex in the local society. Because local opera has strong local characteristics, mixed with various folk cultures, its forms and content are diverse, so local opera is also a more complex folk culture.

### 2.2. The Life Logic of Inheritance

If the “grassroots” artistic characteristics of local opera are formed in the strong local culture, then its orderly inheritance and development between generations depend on the human habitat nurtured by local culture; that is, the traditional farming society has constructed the ideal inheritance field of local opera. During the period of traditional Chinese society, not only did more than three-quarters of the population live in the countryside, but also our cities were “big villages with walls and yamen authorities.” In the vast villages, especially in remote areas, the transportation is inconvenient, the villagers are confined to the closed and small villages to cultivate the land, and life is monotonous. Entertainment, festivals, and sacrifices through opera have become their most convenient and interesting folk activities. In view of the backwardness of the natural economy, the single way of livelihood and the output of farming is not enough to support the family; some people even use singing as a sideline or main means of livelihood to support their families. In addition, the village is a living space based on blood relationships. The villagers live in this “society without strangers,” and they need and are keen to use sound operas to interpret rare legendary stories in daily life. In this way, local opera is deeply rooted in the life of the villagers. Almost every village has a stage. The villagers entertain themselves by “singing opera” during the slack time of farming and during the festivals. For birthdays, weddings, funerals, weddings, and other happy events, every household will invite the troupe to perform a play to celebrate, and singing has become a daily life in rural society. Under this “life-oriented” mechanism, the local people in the popular areas of each local opera can sing and enjoy it, and local opera can be passed down from generation to generation through this “group entertainment practice.”

In the period when local operas were popular, the troupes of local operas spread almost all over the villages. Every time the troupe performs a play, they can get a spontaneous donation from the audience or the bride price of the inviting party. In order to win more performances and good social prestige, each troupe pays attention to its own development. On the one hand, they organize actors to write scripts and strive to diversify the content of performances. On the other hand, they attract artists with superb acting skills to join the troupe, strengthening internal training and improving acting skills. Every artist wants to enter a troupe with a good reputation in order to gain both fame and fortune in terms of economic income and social reputation. They choose a good opera troupe as much as possible and rely on it as an organization for learning and development. There are various ways for actors to learn art. It is the most common and convenient for actors to learn art from apprentices within the troupe, followed by “scoop learning” from peers, and then to improve their acting skills with the help of performance opportunities. Some actors get close to the troupe leader to get all the resources that are beneficial to their own performance development and use this to grow into the “stage pillar” of the troupe, while some actors who grow into the “stage pillar” have set up another troupe to become the troupe leader, seeking personal development of the performing arts career. In this way, the troupe and the actors are interdependent, and they take all the action strategies that are beneficial to their own development and jointly promote the link between the two-the inheritance and the development of local opera. In traditional society, although actors are discriminated against, they are subject to general social and economic poverty. Acting can become a means of earning a living for some lower-class people and even a rare opportunity to be promoted to the upper class of society. Therefore, many children from peasant families have been attracted to opera troupes since childhood. They studied with a teacher and loved their acting career all their life. During the investigation in Guangxi, a provincial inheritor of local opera who was nearly seventy years old told the author that there were 13 friends in the same village who joined the opera troupe with him to learn opera. Acting is a means of earning a living for troupes and actors, and it reflects the “survival” nature of human beings. Under the “survival” mandatory mechanism, local opera has been effectively inherited with the “master-apprentice + performance” model. In cities, the inheritance of local opera mainly depends on various artists and art schools, which attract inheritors to follow them through their own fame.

Field theory holds that the existence of any kind of social space will inevitably generate its habitus so as to ensure the stability and persistence of the field and to discipline the practical subjects in the field. Habitus, once formed, “can generate an infinite, relatively unpredictable, but limited variety of practices” and “ensure the effective existence of prior experience. They have the same characteristics over time.” The continuous existence of the traditional social field and the local field not only reflects the construction of habits but also promotes the lasting role of habits, and the local opera and other folk cultures have developed under the construction of this traditional habit. Therefore, in the traditional field, local opera has always been the choice of local people's pastime and some farmers to make a living. With the practical logic of “living” and “survival,” it enriches the daily life of the public and achieves its own art. 

## 3. Inheritance and Retention of Local Opera

### 3.1. The Inheritance of the Classic Works

Classical works represent the main charm and cultural meaning of local opera, and the inheritance of classic works is the protection of this culture. On May 20, 2006, Guinan Tea-Picking Opera was approved by the State Council of the People's Republic of China to be included in the first batch of national intangible cultural heritage lists. But the drama cannot be a museum art with only text, photos, and video materials. The written record is limited, the photographic record is one-sided, and the image data can have a relatively complete record. But images are “dead” after all, opera is the art of “corner,” and it is the right way to inherit from people. The first problem of inheritance is to retain the most original things of the classic repertoire. Only these orthodox things can have the premise of innovation and development. In the history of development, Guinan Tea-Picking Opera has also continuously integrated other elements of “tea-picking opera” to form what it is today and has also formed a set of program system and performance characteristics that belong to Guinan Tea-Picking Opera and created mature classic works, as shown in Figure 3. It is the imprint of the times in the development of Guinan Tea-Picking Opera, these imprints also need to be preserved as they are, and people (performers) must be preserved together with the video materials [14]. There is a special way of inheritance of opera, which is “oral and heart teaching.” The artistic characteristics of opera “jiao'er” also depend on people. The biggest factor for a classic play to become a classic is the performer's personal skills and the charm of performance style.

### 3.2. Music Features

Guinan selected tea opera, as one of the local classic operas, has many musical style similarities with other “selected tea operas.” “Witty” and “fun” are the two characteristics of the music of Guinan Tea-Picking Opera. First of all, Guinan Tea-Picking Opera and other tea-picking operas are products derived from life. Its melody often appears in tea-picking labor scenes, and this melody has become a way for people to soothe their emotions and regulate fatigue. Most of the stories told in Nancai Tea Opera focus on the trivial life of the common people. The melody of the music is funny and humorous, which brings people a sense of physical and mental pleasure, and gradually becomes an “entertainment necessity” after work and in life [17]. The music development of Guinan Tea-Picking Opera started with the integration of folk minor tunes. The development process had three stages. The first stage only sang folk minor tunes, the second stage integrated a variety of tea-picking melodies for joint singing, and the third stage developed some folk dance music, which gradually formed the current music system. These include “tea-picking lanterns” such as “watching tea tunes” and “picking tea songs.” In the music melody of Guinan Tea-Picking Opera, there is a melody of “Yuduya” as a lining, which has a unique flavor, and the audience is deeply affectionate and widely sung. Therefore, “Yuduya” has become another common name for Guinan Tea-Picking Opera. Because the Guinan Tea-Picking Opera has a unique performance style that emphasizes both singing and dancing, the singing atmosphere is very lively and enthusiastic in the scenes of multiperson performances, and the singing and dancing scenes are more flexible and eclectic. The free expression style and the melody of “Yu Du Ya” with different emotions make the characters more distinct and their emotions more accurate. The musical features of Guinan Tea-Picking Opera “Yu Du Ya” have become the unique musical elements of the opera, which greatly enhanced the artistic charm of the opera. In the inheritance of the music of the tea-picking opera in southern Guinan, these original, witty, and interesting musical elements should be kept intact for a long time.

Opera in different places have different characteristics.  Table 3 lists the characteristics of 10 kinds of opera, including Yue Opera, Peking Opera, and Kunqu Opera.

### 3.3. Belt Inheritance

Belt inheritance is to drive the people around them to participate in the inheritance of traditional culture. The greatest charm of the art of opera is the people because different actors in the same play will show different artistic characteristics (tastes), in terms of both singing and performance. That is where the saying “acting is a play, watching is a human being.” A former opera artist would perform dozens of plays and many hundreds of plays, and the plays they performed have formed their own set of systems. Practice has almost merged tricks with people. This is his understanding of the work, and he has shown his understanding with the skills he is good at, which has been passed down to this day. Now there are fewer and fewer old artists in the tea-picking opera in southern Guinan, which has sent a signal that the number of local operas in China is decreasing year by year, and it is also because of the departure of old local opera artists [18]. The “Several Policies on Supporting the Inheritance and Development of Traditional Opera” implements the “Famous Traditional Opera-Famous Opera Masters Accept Apprentices to Pass on the Arts” plan and supports all types of opera art performance groups, schools, and research institutions at all levels to adopt “One Belt One, One Belt Two” and other methods, teach the essence of opera performance art, and establish a “two-way communication” mechanism between young teachers of opera colleges and young backbones of opera art performance groups to create good conditions for cultivating a new generation of young top-notch talents. Through the investigation of cultural inheritance in the four regions, it is found that the success rate of cultural inheritance in the four regions is more than 30%, as shown in Figure 4.

Although the development history of Guinan Tea-Picking Opera is not as long as Kunqu Opera, Qin Opera, Cantonese Opera, Liyuan Opera, and so on, it is also an inseparable part of the “tea-picking opera system” in Guangxi and even the whole country. As the representative of “Hakka Tea-Picking Opera,” it should be more important to pay attention to its inheritance; otherwise, the cultural loss of Guinan Tea-Picking Opera will be faster [19].

A representative work of the local opera is listed in Table 4.

## 4. The Development of Local Opera

### 4.1. Create New Products and Promote Development

With the continuous improvement of social development and people's living standards, people's requirements for entertainment projects are also increasing. As a local opera with a profound cultural heritage, there is still a lot of room for market development. Bobai Guinan Tea-Picking Opera (Bobai Folk Art Conservation, Inheritance and Development Center, Tea-picking Department), as one of the few literary and art groups in the country that studies and develops Guinan Tea-Picking Opera, shoulders the important responsibility for the development of Guinan Tea-Picking Opera. It is not easy to create works that can promote the development of dramas, and it is even more difficult to make the works keep pace with the times and make the audience like them. There are various types of art that can attract audiences in the art market now. Local operas are “boating against the current” if they do not create new works. Bobai Guinan Tea-Picking Opera has also found a solution to this problem, analyzed specific problems in detail, and found a breakthrough based on regional characteristics according to local conditions. That is, the Bobai Guinan Tea-Picking Opera will first create a small tea-picking opera based on the stories that are happening around people at the moment and often carry out the activity of “sending the opera into the village,” which strengthens the local people's love for the tea-picking opera.

The tea-picking opera in southern Guinan is a very regional type of opera. As a county with the largest population of Hakka in the country, Guangxi Bobai has brought unique advantages to the development of the tea-picking opera in southern Guinan. The Guinan Tea-Picking Opera is an indispensable cultural and entertainment item in the life of the Hakka people, and it is also a common way for the people of Bobai to connect and express their emotions. Bobai Guinan Tea-Picking Opera has created two large-scale Guinan Tea-Picking Opera works in the past three years. The first is the large-scale Guinan tea-picking drama “Green Pearl Girl.” This drama belongs to a new historical drama. The prototype of the story is one of China's top ten beauties, Green Pearl. The work promotes the protagonist's fraternity and dedication and establishes a local character image. Through the performance of the works, the audience can further understand the regional cultural history and enhance the people's national self-confidence. The second part is based on the historical node of the 100th anniversary of the founding of the Communist Party of China, excavating the deeds of Mr. Zhu Xian, the pioneer of Bobai revolution, and creating a large-scale Guinan tea-picking drama “Bagui Pioneer Zhu Xian,” which promotes the importance of deepening the learning and education of the party history. The measure aims to cherish the martyrs, inspire future generations, and educate the majority of party members, cadres, and the masses to appreciate the power of faith. The development of Bobai Guinan Tea-Picking Opera can judge the situation, seize the opportunity of the development of the times, tap the regional culture, further improve and polish it, focus on highlighting the national attributes of the regional culture, continue to improve the works, interpret the high-quality products in a better state, launch the works, and go to the city and the whole district to tour so that the Guinan Tea-Picking Opera can continue to go further and further.

### 4.2. Improve the Environment, Diversify, and Integrate

The rehearsal field is the guarantee for artistic creation, and the theater is the guarantee for the performance of stage works. A professional opera troupe cannot do without the theater and the rehearsal field. The Bobai Folk Art Conservation, Inheritance and Development Center, Tea-Picking Department is the only professional state-run Guinan Tea-Picking Opera Art troupe in Guangxi, which can be called “the first troupe of Guinan Tea-Picking Opera” in China. In this regard, the current head of the group, Lu Guangdong, knows that changing the environment is one of the problems faced by the troupe's development. To make the tea-picking in Guinan revive, it is necessary to bring out works of higher artistic level and return to the audience's attention. As Bobai Guinan Tea-Picking Opera has actively participated in various theatrical performances in counties and cities over the years, it has been recognized by everyone and has gradually increased the influence of Bobai Guinan Tea-Picking Opera. After reviewing the situation, the head of the group raised the issue of upgrading the rehearsal and performance venues and received corresponding policy support. On the basis of the original rehearsal venue, stage lighting and audio equipment was installed to improve the function of the rehearsal venue. Some daily routines can be completed here. The office building was integrated, and three medium-sized practice halls were renovated. Now that the environment has changed, business and supporting development projects have also been added. First, the training business of tea-picking opera is carried out, and training is provided for some fans and teenagers of tea-picking opera; secondly, in addition to the daily training of actors, the practice hall will also open some singing and dancing classes. It is very important for the development of Bobai Guinan Tea-Picking Opera to better promote the development of this opera to further study how to diversify and integrate development.

### 4.3. Strengthen Talent Training and Establish New Models

No matter what the cultural system is, strengthening talent training is always a major issue. If Bobai Jinan selected tea drama wants to develop better, it is necessary to start from the cultivation of actors. According to the survey, the specific age distribution of the actors in the selected tea drama is shown in Figure 5. The development of local opera should pay attention to the cultivation of young talents and restore the “hematopoietic function.” The development of Bobai Guinan Tea-Picking Opera must start from the cultivation of talents. There must be people for development. Head Lv Guangdong also found a way to develop people and retain people and other issues and formulated a 5-year talent training plan. It is expected to complete the training target of 300 people. The students recruited each year are jointly trained with Guangxi Art School. It is guaranteed to train 50–60 students every year, gradually expand the talent echelon of Bobai Guinan Tea-Picking Opera, and develop the performance team of Bobai Guinan Tea-Picking Opera in the direction of refinement, high quality, and elite. The personnel echelon implements classified management and is divided into Guinan tea-picking team, children's art training team, and singing and dancing performance team. The integration and development of Nancai Tea Opera will continue to broaden the future development path; the establishment of a singing and dancing performance team has enriched the types of performances of Southern Guinan Tea Opera and can also connect commercial performances and cultural tourism performances, gradually making Bobai Guinan Tea Opera a professional and diverse stage performance. 

## 5. Conclusion

Traditional opera has been developed for thousands of years. Today, when various modern entertainment forms such as film, television, and the Internet are booming, various artistic activities are widely carried out, and people have more and more space to choose entertainment forms and art appreciation categories. Under the circumstances, its inheritance has encountered unprecedented difficulties, and a large part of local operas have reached an endangered and lost situation, resulting in the movement of people and the dissolution of groups. Therefore, the protection and inheritance of traditional opera cannot rely solely on cultural workers.

Through the analysis of local opera cases, especially the development of local opera and music, this paper tries to solve the inheritance dilemma and proposes the strategies of creating new products, promoting the development, realizing diversification, integrating resources, strengthening talent training, and establishing new models. This paper is important to developing and promoting the practice of Chinese traditional culture in the same research form in the future [20].

## Figures and Tables

**Figure 1:** Ways that people understand the traditional culture.

**Figure 2:** The top five most popular local dramas on Douyin.

**Figure 3:** Choose the classic elements from the tea play.

**Figure 4:** Success rate of belt style cultural inheritance.

**Figure 5:** The age proportion of the actors selected in tea dramas.

**Table 1:** The national intangible cultural heritage project.

Traditional handicraft skills	Herbal tea making skills, 2006
	Oolong tea making skills (Wuyi rock tea making skills, 2006; Tieguanyin making skills, 2008)
	Black tea making skills (Qimen black tea making skills, 2011)
	Green tea making skills (West Lake Longjing, Aoyuan Juyan, Gongshan Maofeng, Taiping Houkui, and Lu'an Guapian, 2008; making skills of Biluochun, Anji white tea, and purple bamboo shoot tea, 2011)
	White tea making skills (Fuding white tea making skills, 2011)
	Pu'er tea making skills (Gong tea and Dayi tea making skills, 2008)
	Black tea making skills (making skills of Qianliang tea, Fuzhuan tea, and Nanlubian tea, 2008; making skills of Xiaguantuo tea, 2011)
	Flower tea making skills (Zhang Yiyuan and Jasmine tea making skills, 2008; Wu Yutai and Jasmine tea making skills, 2011)
	Refreshment making skills (Fuchun, 2008)

Social customs, etiquette, and festivals	Tea art project: Chaozhou Gongfu tea art, 2008; temple fair project: Gancha farm in Pan'an County, Zhejiang Province, 2008; Jingshan tea banquet, 2011 in Hangzhou, Zhejiang Province
	Chashan Haozi, Chenxi County, Hunan Province, 2008

Performing arts	Gannan Tea-Picking Opera, Guinan Tea-Picking Opera, and Yangxin Tea-Picking Opera, 2006; Gao'an Tea-Picking Opera, Fuzhou Tea-Picking Opera, and northern Guangdong Tea-Picking Opera, 2011

**Table 2:** The influence of a certain local drama on the volcano video.

No.	Volcano nickname	Total number of fans	Firepower	Total number of live broadcasts	Total number of works
1	Taikang Daoqing Li Yanling	2.5 w	4.5 w	68	164
2	Taikang Daoqing Li Yanling	6.5 w	3.4 w	13	1637
3	Taikang Daoqing Art Conservation and Inheritance Center	2094	102	0	24
4	Taikang Daoqing Liu Fanxia	3844	7703	13	919
5	Taikang Taoism Liu Fanxia	2.0 w	4444	27	137
6	Taikang Daoqing Luo Ali	7672	9345	9	332
7	Sun Xiangang	905	2538	25	649
8	Liu Xiuwu	37	7	0	3
9	Zong Xiankun	62	337	0	58
10	Huibao	1.3 w	1.7 w	81	412
11	Dodo	4.2 w	3.8 w	118	1707
12	Zhang Xiaoyu	1.6 w	2.3 w	9	410
13	Bright	1.3 w	1.7 w	66	1837
14	Daoqing Xiaojun	4549	1.2 w	62	1140
15	Taikang Daoqing Zhang Lei	2263	5563	28	787
16	Zhang Feng	112	271	0	92
17	Taikang Daoqing Pear Orchard Chun Lei Luo Aihua	117	380	2	106
18	Hou Zhenzhen	2.2 w	3.0 w	64	150

**Table 3:** Features of ten local operas.

Species	Characteristics	Main regions
Yue Opera	Lyric, with a clear and graceful voice, beautiful and beautiful, and the performance is real and moving, with a strong Jiangnan local color	Zhejiang, Shanghai, Jiangsu, Jiangxi, Anhui, and Fujian
Henan Opera	The voice may be high and lively or sad and lingering	The vast northern areas of the Yellow River and Huai River Basin
Pingju	The articulation is clear, the singing is clear, and the performance is full of life, lively, and free	Beijing, Tianjin, Hebei, and the three northeastern provinces
Kunqu Opera	Strong lyricism and delicate movements	Jiangsu, Shanghai, Zhejiang, and Beijing
Huangmei Opera	Beautiful melody and a touching story and having a wide range of influence on people	Anhui, Jiangxi, and Hubei
Sichuan Opera	Miscellaneous and diverse voices	Sichuan, Chongqing, Guizhou, and Yunnan
Jin Opera	High-pitched but also soft and delicate	Shanxi, Inner Mongolia, Shaanxi, and Hebei
Hebei Bangzi	High-pitched and passionate singing, generous, compassionate, melodious, and melodious	Central and Northern Hebei and Beijing-Tianjin area
Qin Opera	The voice is deep, mournful, and impassioned, and the voice is cheerful, lively, strong, and powerful	Northwest region
Cantonese Opera	Diverse and expressive	Guangdong, Guangxi, Southern Fujian, Hong Kong, and Macau

**Table 4:** Representatives of local operas.

Type	Representative
Yue Opera	Yuan Xuefen; Xu Yulan
Henan Opera	Chang Xiangyu; Wang Xiulan
Pingju	Li Jinshun; Moon Pearl
Kunqu Opera	Liang Chenyu; Tang Xianzu
Huangmei Opera	Yan Fengying; Han Zaifen
Sichuan Opera	Jia Peizhi; Zhou Mulian
Qin Opera	Ma Youxian; Pan Zonghan
Cantonese Opera	Xue Juexian; Ma Shizeng

## Data Availability

The labeled data set used to support the findings of this study is available from the corresponding author upon request.
